# Comparison of Idiopathic Macular Hole Interventions Using Frequency Domain Optical Coherence Tomography and Optical Coherence Tomography Angiography

**DOI:** 10.1155/2022/7749605

**Published:** 2022-08-13

**Authors:** Miao Liu, Yu Jin, Liu Li, Fangxiu Yuan, Yueyuan Xu

**Affiliations:** Ophthalmology Department, The First Hospital of Nanchang, NanChang, China

## Abstract

**Objective:**

We aimed to determine the efficacy of different idiopathic macular hole treatment methods to improve recovery time and patient outcomes using Frequency Domain Optical Coherence Tomography (SD-OCT) and Optical Coherence Tomography Angiography (OCTA).

**Methods:**

This retrospective study included patients with idiopathic macular hole who were admitted to our hospital between 1st January 2019 and 31st October 2021. The control group was treated with internal limiting membrane tamponade, and the study group was treated with clamshell therapy. Treatment conditions (internal limiting membrane treatment duration and hole closure rate), best corrected visual acuity (BCVA) before and after surgery, OCTA measurements, and SD-OCT were assessed. The retinal nerve fiber layer (RNFL), retinal ganglion cell layer (GCL), and retinal pigment epithelium (RPE) thicknesses were also analyzed.

**Results:**

The treatment time and hole closure rate of the internal limiting membrane in the study group were higher than those in the control group. The curative effect of the study group was better than that of the control group. The postoperative DCP blood vessel density in both groups was higher than that before operation, and the study group was higher than the control group. The FAZ area and circumference were lower than those before surgery, and the study group was lower than the control group. At 3 months after operation, the thickness of DIOA, nasal temporal RNFL, and GCL were decreased in both groups, and the observed values in the study group were lower than those in the control group. At 3-month follow-up, there was no significant difference in RPE thickness between the two groups.

**Conclusion:**

Flip and cover therapy is the most effective treatment. SD-OCT and OCTA provide an objective basis for clinical intervention by comparing the effects of different procedures on the retinal condition of patients.

## 1. Introduction

Idiopathic macular hole refers to a macular hole spontaneously occurring for reasons other than fundus disease, resulting in severe damage to patients' central vision [1]. Removing the vitreous cortex when treating idiopathic macular hole and peeling the internal boundary membrane near the hole eliminates horizontal traction on the hole margin, resulting in closure of the hole. However, among those with refractory macular hole (large diameter hole and high myopia), patients with low hole closure rates are prone to irregular closure morphology, which affects visual function recovery [2, 3]. Therefore, treating idiopathic macular hole safely and effectively is of great importance.

Internal limiting membrane tamponade and partial stripping of the internal limiting membrane after the remaining internal limiting membrane flip cover are commonly used in clinical improvement, which can promote cell proliferation and reconstruction of foveal structure, avoid contact with the vitreous lumen material of the exposed outer retina, and improve the rate and morphology of hiatus closure [4, 5]. Frequency Domain Optical Coherence Tomography (SD-OCT) and Optical Coherence Tomography Angiography (OCTA) can determine the fine structure of macular area before and after the operation in patients with idiopathic macular hole so as to provide a reference basis to evaluate the effects of the operation [6, 7].

Based on the abovementioned facts, we attempted to analyze and discuss the application value of SD-OCT and OCTA to evaluate the effect of different idiopathic macular hole operation methods.

## 2. Materials and Methods

### 2.1. Baseline Data

This retrospective study included the patients with idiopathic macular hole who were admitted to our hospital between 1st January 2019 and 31st October 2021. The protocol of this study was approved by the ethical committee of the first hospital of Nanchang.

### 2.2. Inclusion and Exclusion Criteria

The inclusion criteria were as follows: (1) idiopathic macular hole was diagnosed using slit lamp enteroscopy and three mirror gonioscopy before the procedure, (2) idiopathic macular hole in only one eye, (3) idiopathic macular hole stages II-IV, and (4) informed consent of patients and their families. The exclusion criteria were as follows: (1) diabetic retinopathy, (2) cataract nucleus above grade IV, (3) age-related macular degeneration, (4) retinal detachment, (5) history of fundus surgery, and (6) history of ocular trauma.

### 2.3. Methods

Patients in both groups underwent standard three-port, planar vitrectomy, and filling with disinfected air or silicone oil. After removing the central visual axis vitreous via vitrectomy, artificial posterior vitreous detachment was performed to ensure the complete removal of the posterior vitreous cortex. Bright blue staining showed the morphology of the internal limiting membrane. The internal limiting membrane was moved approximately 1 PD away from the fovea, and the stripping range extended to ≥2 PD. In the study group, one side of the internal limiting membrane was removed while the remaining side of the internal limiting membrane was used to cover the hole. In the control group, the inner limiting membrane of the remaining annular fovea was released and used to fill the fissure. If the internal limiting membrane is not easily fixed in the vitreous cavity due to its high mobility after release, a small amount of heavy water should be used to flatten it. After gas-liquid exchange, the vitreous cavity was filled with intraocular gas or silicone oil.

### 2.4. Observation Indexes

The following parameters were determined in this study: (1) treatment status (internal limiting membrane treatment time, hole closure rate), (2) best corrected visual acuity (BCVA) observed before and after surgery, (3) preoperative and postoperative results of density, area, and circumference of OCTA superficial capillary plexus (SCP) and deep capillary plexus (DCP) using OCT (RS-3000 Advance, NIDEK) to measure foveal avascularity, and (4) SD-OCT measurement results before and after surgery (photoreceptor inner and outer ganglion deletion zone (DIOA), retinal nerve fiber layer (RNFL), retinal ganglion cell layer (GCL), retinal pigment epithelium (RPE) (horizontal diameter) thickness) were obtained using SD-OCT (Topcon version 3.21) [8, 9].

### 2.5. Statistical Methods

The SPSS 21.0 software (IBM, Chicago, USA) was used to analyze data. Measurement data was expressed as mean ± *s* and was evaluated using the *t*-test, while enumeration data was expressed as *n* (%) and analyzed using the *χ*^2^ test. The two-sided *P* < 0.05 indicated a statistically significant difference.

## 3. Results

### 3.1. Treatment Conditions

A total of 94 patients were included in this study. The patients' gender distribution, age, body mass index, location, hiatus diameter, and stage in each group were similar, as shown in Table 1. The duration of treatment of the internal limiting membrane and hiatus closure rate of the study group was higher than that of the control group, and the difference was statistically significant (*P* < 0.05), as shown in Table 2.

### 3.2. Best Corrected Visual Acuity

The BCVA between the two groups did not differ significantly before the procedure (*P* > 0.05), while the BCVA of both groups was improved at 1 month and 3 months after the operation compared to that before the operation. The study group exhibited better outcomes than the control group, and the difference was statistically significant (*P* < 0.05), as shown in Table 3.

### 3.3. OCTA Measurement Results

The groups did not differ significantly in terms of SCP and DCP vascular density, FAZ area, or circumference before the procedure (*P* > 0.05). After the operation, the DCP vascular density in both was higher than that observed before the procedure. That of the study group was higher than that of the control group. The area and circumference of FAZ were lower than that observed before surgery, and that of the study group was lower than that of the control group (*P* < 0.05). SCP vascular density did not differ significantly between the two groups (*P* > 0.05), as shown in Table 4.

### 3.4. SD-OCT Measurement Results

The DIOA, nasal and temporal RNFL, GCL, and RPE thickness measurements did not differ significantly between the two groups before their respective procedures (*P* > 0.05). The DIOA, nasal and temporal RNFL, and GCL thickness had decreased three months after surgery in both groups, and the measurements of the study group were lower than those of the control group. The difference was statistically significant (*P* < 0.05). No significant difference in RPE thickness was observed between the two groups at a three-month follow-up (*P* > 0.05), as shown in Table 5.

## 4. Discussion

Vitreous dissection of the internal membrane has become the standard of treatment among cases of idiopathic macular hole. Most idiopathic macular holes heal well, and visual function may improve due to internal boundary membrane dissection alone [10]. However, for holes with a large diameter (>600 *μ*m) and refractory macular holes with high myopia, the effect of internal boundary membrane stripping on the healing state of the hole and the improvement of visual acuity is not satisfactory [11]. Blindly expanding the scope of inner boundary membrane stripping and minimizing the horizontal traction of the hole are not the best means to treat these cases, as this can easily result in a large portion of the retina being exposed (lack of inner boundary membrane coverage). In addition, according to a recent anatomical study, these methods can cause Müller cell injury, optic nerve fiber layer detachment, temporal retinal thinning, macular displacement, and other complications [12, 13]. Meanwhile, vertical vitreous traction of the pore margin causes retinal structural damage, a large amount of contact between the outer retina and vitreous lumen materials, and edema of the pore margin, resulting in the apoptosis of Müller cells, especially in patients with refractory macular hole [14]. In China, which has a large population base and an increased incidence of high myopia, there are several patients with refractory macular hole. Therefore, improving the outcomes of inner boundary membrane stripping is vital.

Internal limiting membrane tamponade, as well as overturning and covering, was recently proposed as methods to improve internal limiting membrane dissection, which can prevent some of the adverse consequences of removing the internal limiting membrane. These are also effective means to treat refractory macular hole [15, 16]. Intermedial membrane tamponation uses the remnants of the intermedial membrane as a scaffold to induce retinal glial cells to enter the macular foramen and stimulate photoreceptor cell migration and Müller cell proliferation, thereby strengthening hiatus closure [17]. The holes were closed during the operation to prevent the outer retina from making contact with the filling material in the vitreous cavity, which may inhibit the hydration of retinal tissue, maximize the preservation of Müller cells in the retina around the holes, increase the elasticity of the inner retina, promote the centripetal movement of the retina and active reconstruction of the fovea structure, and improve visual function [18, 19]. Our results indicated that the BCVA and the closure rate of hiatus in the study group were higher than those of the control group when measured 1 and 3 months after the operation. The differences were statistically significant (*P* < 0.05), indicating that overturning and coverage can improve the visual function of patients with idiopathic macular hole more effectively and improve the hole closure rate. Gaber et al. [20] also found that the hiatus closure rate was higher than that of patients with internal boundary membrane tamponade, but the improvement of visual function was similar between patients who underwent the two methods. This study differed in that the recovery of visual function was related to the degree of retinal choroid atrophy and the time of existence of the hiatus, which varies greatly. However, the treatment time of the internal boundary membrane during the reversal and overlay was long, which is due to the complicated nature of reversal and overlay and the increased difficulty of the operation.

In the present study, OCTA was used to compare measurements of the FAZ area, circumference, and retinal circulation in the macular area before and after the operation. The area and circumference of FAZ in the study group were lower than those of the control group 3 months after the operation (*P* < 0.05). This may be because the removal of the inner boundary membrane improved retinal surface flexibility and the peripore tissues were concentrated in the fovea. Meanwhile, the macular tissue structure recovered after the operation, and the recovery effect of overlay improved. In patients with idiopathic macular hole, stratified cysts surround the hiatus, and DCP is mainly located between the inner and outer plexus layers. The cysts in this layer are large, elongated, and radiating and exhibit reduced vascular density. Our data showed that the vascular density of DCP in the two groups was higher 3 months after the operation than that before the operation, because the cystic cavity around the macular hole disappeared after operation and the blood flow density increased. Moreover, the vascular density of DCP in the study group was higher than that in the control group, which may be related to better retinal recovery after turnover covering.

SD-OCT is a recently developed technology. The 10-layer retinal structure can clearly be identified due to its high resolution; thus, it can detect retinal and macular disease at a sensitivity level similar to that of histopathology. The image can also be taken quickly to avoid the artifact of eye movement [21]. The integrity of the IS/OS layer is an important indicator of photoreceptors' integrity [22]. It is an objective and repeatable index that measures the maximum DIOA value between the breakpoints of IS/OS connection lines. The present study demonstrated that DIOA had decreased significantly in both groups 3 months after the surgery and that the values of the study group were significantly lower than those in the control group (*P* < 0.05), suggesting that overlaying could mitigate the damage to the IS/OS layer more effectively in patients with idiopathic macular hole. This is because roll-over coverage results in the maximal preservation of Müller cells in the retina, promotes hiatus closure, treats retinal edema, and thus mitigates the IS/OS layer damage more effectively. Retinal ganglion cells are the most vulnerable to retinal ischemia and inflammation. The data of the present study showed that both groups' nasal and temporal RNFL and GCL thickness decreased significantly 3 months after the operation, and the values observed in the study group were lower than those of the control group (*P* < 0.05); therefore, flip and cover therapy is a better treatment for retinal edema.

## 5. Conclusion

Flip and cover therapy has a high application value in the treatment of idiopathic macular hole, and the retinal recovery and hole closure rates in the study group were better than those observed in the control group. SD-OCT and OCTA examination can elucidate the effect of different operations on the patients' retinal condition to provide an objective reference basis to plan a clinical intervention.

## Figures and Tables

**Table 1:** The comparison of baseline data between the two groups.

Data	The study group (*n* = 47)	The control group (*n* = 47)	*t*/*χ*^2^	*P*
Gender (male/female)	19/28	17/30	0.180	0.671
Age (years old)	49~76 (61.75 ± 4.97)	47~79 (63.04 ± 5.28)	1.220	0.226
BMI (kg/m^2^)	18~29 (21.95 ± 1.79)	17~30 (22.19 ± 1.92)	0.627	0.532
Location				
Left eye	25 (53.19)	27 (57.45)	0.172	0.678
Right eye	22 (46.81)	20 (42.55)		
Hiatus diameter (*μ*m)	430~690 (586.74 ± 45.63)	415~695 (591.37 ± 47.28)	0.483	0.630
Stage				
Stage II	11 (23.40)	12 (25.53)	0.173	0.917
Stage III	22 (46.81)	20 (42.55)		
Stage IV	14 (29.79)	15 (31.91)		

**Table 2:** The comparison of treatment conditions between the two groups.

Groups	Cases	The treatment time of internal limiting membrane (s)	Closure rate of hiatus, *n* (%)
The study group	47	625.38 ± 55.42	43 (91.49)
The control group	47	449.47 ± 46.53	35 (74.47)
*χ* ^2^/*t*		16.666	4.821
*P*		0.001	0.028

**Table 3:** The comparison of best corrected visual acuity between the two groups.

Groups	Cases	Before the operation	1 month after the operation	3 months after the operation
The study group	47	1.50 ± 0.13	1.07 ± 0.15	0.85 ± 0.10
The control group	47	1.48 ± 0.12	1.20 ± 0.16	0.94 ± 0.12
*t*		0.775	4.064	3.950
*P*		0.440	0.001	0.001

**Table 4:** The comparison of OCTA measurement results between the two groups.

Time	Groups	Cases	SCP vascular density (%)	DCP vascular density (%)	FAZ	
					Area (mm^2^)	Circumference (mm)
Before the operation	The study group	47	11.85 ± 3.51	13.86 ± 3.72	0.57 ± 0.15	2.59 ± 0.47
	The control group	47	12.09 ± 3.82	14.59 ± 3.51	0.60 ± 0.17	2.64 ± 0.53
	*t*		0.317	0.979	0.907	0.484
	*P*		0.752	0.330	0.367	0.630

3 months after the operation	The study group	47	11.63 ± 3.47	21.05 ± 4.14^a^	0.35 ± 0.13^a^	1.59 ± 0.28^a^
	The control group	47	11.84 ± 3.65	16.93 ± 4.05^a^	0.47 ± 0.14^a^	1.97 ± 0.36^a^
	*t*		0.286	4.877	4.306	5.712
	*P*		0.776	0.001	0.001	0.001

Note: compared with the same group before surgery, ^a^*P* < 0.05.

**Table 5:** The comparison of SD-OCT measurement results between the two groups.

Time	Groups	Cases	DIOA	RNFL		GCL		RPE	
				Nasal	Temporal	Nasal	Temporal	Nasal	Temporal
Before the operation	The study group	47	1893.25 ± 246.84	33.45 ± 0.96	21.15 ± 1.76	49.58 ± 2.76	42.75 ± 2.57	13.10 ± 1.79	15.81 ± 1.93
	The control group	47	1936.87 ± 302.48	33.61 ± 1.05	20.95 ± 1.58	50.04 ± 3.15	43.12 ± 2.83	12.93 ± 1.85	16.07 ± 2.06
	*t*		0.766	0.867	0.580	0.753	0.664	0.453	0.631
	*P*		0.446	0.388	0.564	0.453	0.509	0.652	0.529

3 months after the operation	The study group	47	1297.54 ± 225.61^a^	30.09 ± 0.89^a^	18.25 ± 1.39^a^	38.35 ± 2.94^a^	25.16 ± 2.28^a^	12.95 ± 2.04	15.53 ± 2.17
	The control group	47	1504.61 ± 275.58^a^	31.54 ± 1.12^a^	19.41 ± 1.28^a^	40.63 ± 3.07^a^	28.05 ± 2.47^a^	13.04 ± 1.92	15.79 ± 1.85
	*t*		3.986	6.949	4.208	3.677	5.894	0.220	0.625
	*P*		0.001	0.001	0.001	0.001	0.001	0.826	0.534

Note: compared with the same group before surgery, ^a^*P* < 0.05.

## Data Availability

Data is available upon request.
